RETRACTED

# Building Interior Layout Design Based on Building Information Model and Deep Learning Technology: Taking the Interior Renewal Design of the Fifth Floor of the Procuratorate of Dong Xi Hu District as an Example

**DOI:** 10.1155/2022/3746393

**Published:** 2022-10-10

**Authors:** Haowei Pan, Gewei Zheng, Ákos Hutter, Zhenkai Huang

**Affiliations:** ^1^Faculty of Engineering and Information Technology, University of Pecs, Pécs, Hungary; ^2^School of Art & Design, Hubei University of Technology, Wuhan, China

## Abstract

With the development of the Internet era and the information age, electronic information technology has profoundly affected human life and work, and the architectural design industry is no exception. Architectural design has a complex design period, and the arbitrary division of labour reflects the particularity of its working process. At present, the integration of electronic information technology and scientific and technological software into architectural design has dramatically improved the work efficiency of designers. However, due to the enormous workload of drawing and modification of building drawings, and many professional departments involved in cooperation, the error rate of drawing design is still high, which eventually leads to a series of serious problems such as stagnation of the design process and rework of construction. However, due to the enormous workload of drawing and modification of building drawings, and many professional departments involved in cooperation, the error rate of drawing design is still high, which eventually leads to a series of serious problems such as stagnation of the design process and rework of construction. The BIM building information model system is an electronic information platform for comprehensive architectural design majors. It can integrate the design drawings of various majors in the design process, correct the design problems caused by inaccurate pictures at the first time, and reduce the errors in the design process. Through the BIM system and Python programming software, cross-platform cooperation is carried out to carry out computer deep learning and a series of extra design work. This paper puts forward the interior design method of the BIM system and shows the research work of interior design by the BIM building information platform through practical cases. By comparing with traditional design methods, the advantages of this technology in interior design are demonstrated, and a reference for future interior design informatization is provided.

## 1. Introduction

The development stage of the interior design project includes the conceptual design, scheme design, construction design, construction documents, procurement, construction management, and operation and maintenance. It is used to manage the project to show the McClam curve (Figure 1). The *X* axis is the stage of the design project. The *Y* axis shows the effect value of each step. The cost changes brought by the change of time in each stage of the curve design. The figure shows that in the later stage of the project, the project cost caused by any design change will increase sharply. Therefore, we can conclude that the earlier the design phase is completed, the less modification and the less cost of the project will be required.

RETRACTED

Nowadays, the vast majority of Chinese interior design companies through two-dimensional design software “*CAD*” and three-dimensional modelling software and rendering software (*3dmax*, *sketch up*, *Lumion*, and *V-ray*) combined with the actual operation of the design project (Figure 2).

Although the combination of 2D design software and 3D design software solves the problem of file attenuation [1] during transmission to a certain extent, this method of information transmission has the problems of low efficiency, poor information coordination and sharing, and its files are purely computer-drawn spatial models. They cannot convey all the information required by different work departments. With China's building informatization, although the building information rate has gradually developed steadily, the current design informatization rate is only 0.03%, which is a huge gap compared with the international average of 0.4%. The efficiency of design information transfer has become the main reason for the low efficiency of design and construction production [2]. With the gradual use of the electronic information technology of Python computer learning software technology, the design project information should become more complete and in-depth. However, most of the research at home and abroad focuses on the technical optimization concept scheme [3], and they ignored the process of how the concept of interior architects was generated and did not explore the possibility of deep learning in the generation stage of architectural plans, resulting in a low degree of fit between the proposed solutions and interior plan designers, and the system was too abstract to be applied [4]. Based on the problem, this paper attempts to study the learning method of interior design concept generation driven by the BIM system and Python deep learning platform, assisting designers in preliminary design, improving design efficiency, and complete information transmission.

### 1.1. Information Logic Based on the BIM and Python Platform

In addition to the influence of personal aesthetics, there are many other constraints in the design stage, such as regional functions, style elements, material types, and the type of environment where the project is located. These conditions need to be reflected in the design results, which will ultimately affect the final outcome of the design scheme. The article calls the condition-constrained [5] design generation rule “experience element.” The concept scheme of interior design synthesises the results of design logic training and design element trade-offs. Although design tasks are different, the design logic principles are almost identical. According to the existing rules and conditions, combined with professional knowledge and design experience, the designer finally obtains the design results. Using the principle of the mapping function, it can be recorded as Fe: [F(xc)⟶G(xs)], where F(xc) is the set of design conditions, *G*(xs) is the set of design concepts, and Fe is the experience factor [6].

RETRACTED

### 1.2. Information Logic Based on the BIM Platform

When the mathematical logic is correct, how correctly extracting the internal contour of the building is particularly important for interior design, and it is also the first step to obtaining architectural information. It comes from two-dimensional architectural drawings, photos, or IFC building information model. The first two need to be manually identified, and the third can be automatically obtained by BIM software. IFC (industry foundation class), as a general information transmission format of BIM software, can be used as an information extraction source for interior design planes, as shown in Figure 3.

### 1.3. Pretreatment of Building Plan

The building's inner wall and frame column are the basis for determining the indoor contour, so the purpose of image preprocessing is to highlight the area of the inner wall and the column between the walls. Its advantage is improving image recognition accuracy and reducing computational complexity.

Firstly, the BIM information model is generated according to the architectural contour map of the East-West Lake District Inspection Institute in Wuhan City, Hubei Province, drawn by the author, and then the internal space of the building is stripped out to generate solid polygons. In order to simplify the subsequent design process, the internal contour map of the building is filled with a red and green background, and the image is generated. Finally, the drawing is binarized. The process is shown in Figure 4.

## 2. Technical Features of Deep Learning in Solving Design Problems

As a method to realize artificial intelligence, the logic of deep learning is that computers parse data files through mathematical formulas and algorithms and make decisions through data learning. Its essence is computer anthropomorphic learning technology [7]. The computer algorithm simulates the creative steps of designers in the design scheme period, finds the potential laws of designers in the design process, and conducts computer learning through the rules, to help designers better complete the design work in the design process. Design steps have the following similar steps.

RETRACTED

### 2.1. Case Study

This step is the process in which designers use past practice cases or similar cases to predict the current scheme [8], which can also be called the database of the designer. The core of deep learning is to establish the corresponding learning group or database through learning evidence, learn and dig data repeatedly through the input layer and output layer of python, and finally obtain the ability to solve problems.

### 2.2. Experiential Learning

As mentioned above, the role of deep learning is to simulate the designer's daily work and learn to assist the designer's work, that is, to get the same or similar practical experience with the designer, and then screen out used cases and expertise for design, for accurate design projects.

### 2.3. Design Ability

Through the continuous strengthening of experience ability, interior designers can strengthen their ability to control different schemes and project landing. In short, the more design knowledge and practice case reserves, the more accurate the design of the designer and the more in line with customer expectations. Similarly, the more the number of deep learning training, the more consistent with human behaviour and the ability to solve design problems closer to the real solution [9].

Therefore, the design process of the scheme design is based on the possibility of expected verification of the design results made by indoor designers according to the control factors of the project. This is the problem that deep learning is good at solving and the key that this technology can be used to solve similar problems.

## 3. Space Generation Experiment Based on Actual Project

In summary, this paper attempts to propose a method based on the BIM information technology model and Python deep learning and proposes the generation method of an interior design scheme. This method combines the advantages of complete design information of the BIM information technology model and the intuitive benefits of python code and obtains the generation results of interior design by simulating and learning the design process of the designers (Figure 5).

The premise of any spatial generation behaviour is to obtain the design background information and design basis. According to the solid design background, the author describes the project as follows:

RETRACTED

### 3.1. Background of the Project

*Dong Xi Hu* District (Figure 6) is located in the west of Wuhan. The area is about 495 km^2^, with 11 streets and an urbanization rate of 63.28% [10].

The procuratorate building is located in Erya Road, Dong Xi Hu District, Wuhan city (Figure 7). The building is an important government function in East-West Lake District. The design team aims to provide a more functional and flexible space for the office space design of the fifth floor of the office building of the public prosecutor's office without damaging the main structure of the building, improve the original organizational structure of the building space, and enhance the user's office efficiency and office experience. Different ages have created different design thinking, aesthetic standards and functional requirements, and the building has a series of life processes such as development, functional degradation, and renewal from the beginning of construction, which is a developing dynamic object [11]. Therefore, the space transformation of buildings is essentially a supplement to the process of building life so that the old buildings better match today's working environment. Modern office or life is looking forward to a new type of plane for indoor planning [12]. The function of the interior design is not only to divide the interior space of the building reasonably but also to combine the function and aesthetics to provide users with a good and comfortable working and living environment. The building of the East-West Lake District Procuratorate was completed around 2000. The office area on the fifth floor is mainly office space, lacking sizeable public space. In today's working environment, single-room-based office buildings lead to a small span of office buildings, narrow and blocked indoor space, which is not conducive to the modern office, and even causes the user's heart depression [13]. Modern office mode is an office mode with high strength and high openness. To meet the new mode of contemporary office, it is necessary to break the barriers between offices as much as possible in interior design and create a transparent and spacious office environment to promote the communication of office workers. *Jan Gehl* mentioned in the communication space that “improving the conditions of activities in public space will indirectly promote the social activities of the users” [14]. Due to the internal structure of the building, there are some problems to be solved in the field space. The author found the following issues through field research.

#### 3.1.1. Lack of Public Space

Due to traditional Chinese design thinking, the interior space of government office buildings (Figure 8) is dominated by single rooms [15]. The essence of this design thinking is to privatize public space, forming closed personal or departmental spaces. They can only stay in their respective offices during work and cannot communicate with other colleagues.

RETRACTED

#### 3.1.2. Lack of Leisure Space

Functionality, practicability, and aesthetics are the three principles of architecture [16], and buildings' external and internal forms must be within the framework of the three principles. The single room and aisle constitute the main body of the interior space of the building on the 5th floor of the Dong Xi Hu District Procuratorate. However, due to the singleness of the internal structure of the procuratorate, there is a lack of a certain amount of leisure space, which eventually leads to the single internal function of the procuratorate, and the lack of vitality inside the building.

### 3.2. Design Generation Process

The author uses design methods such as literature collection, data sorting, and machine operation, combined with on-site research, design requirements, and design room types in the office area and concludes that the types of rooms that may appear in a dynamic office space can be summarized as Table 1.

The author defines the principle of rule combination of modules of basic room and particular room. Different splicing results will appear due to different room splicing. In order to avoid design logic errors and to learn confusion, it is necessary to customize an evaluation system as shown in Table 2, before deep learning [16–20]. The specific room usage is formulated according to the design task book, the connection relationship between the rooms in the building follows the principles of interior design and basic common sense, such as the connection between the office and the corridor, and the connection between the coffee shop and the corridor, which is used to judge the design logic of the identification result of the office space.

### 3.3. Experimental Results

Generation experiments chose using the NetworkX [21–26] network package. NetworkX is a network modelling tool developed based on the python platform. Its connotative network analysis method can provide users with network analysis and modelling of building planes [27–29]. NetworkX includes storing image classes, creating image classes, and implementing image drawing functions through the Graphviz [18] tool library. The experimental platform of this interior design scheme generation experiment is Dell G15, the operating environment is Windows 10, the CPU core is AMD Ryzen5800H octa-core, the physical memory is 16 GB, and the graphics card is GeForce GTX3060. The experiment is based on the design scheme plane for the generation (Figure 9).

RETRACTED

Using the NetworkX toolkit [30–32] and the constraints in Tables 1 and Table 2, the author defines the room type and spatial link as corridor link and door link. The program is mainly as follows:

  Import networks = nx
  G = nx,graph
(1) G = add_node(floor = 1,type = “corridor”)
  G = add_node(floor = 1,type = “office”)
  G = add_node(floor = 1,type = “coffee-room”)
  G = add_node(floor = 1,type = “meeting-rooms”)
  G = add_node(floor = 1,type = “library”)
  G = add_node(floor = 1,type = “relax spaces”)
  G = add_node(floor = 1,type = “prsecutor's museum”)

Add _ node ( ) is used to create connection nodes. The author defines ten as the first node number, and the second parameter floor is defined as the floor. Since the design area is the same floor, namely floor = 1. The type is defined as the room type parameter. At the same time, two connection modes of the door and corridor are defined. After the establishment is completed, the nx drawn ( ) equation is called for visual editing, and then the topological graph is obtained (Figure 10). The region-linked bubble map is generated from the existing base map.

Finally, the concept of interior design graphic is generated in the new design area (as shown in Figure 11), and the equation is visually edited by nx and drawn to obtain the new topological graph. Under the premise of determining the appropriate functional link, the effectiveness of the design block splicing is manually determined, and then BIM software is used to convert the plane drawings that can be used by designers. The plane drawings that can be used by designers are shown in Figure 12.

## 4. Conclusions

The combination of deep learning and interior design has broad prospects. Its appearance can not only simplify the complex and repetitive work of designers in the early stage of design but also generate design plans through neural network learning and achieve the automatic design. Some companies' copywriting work already accomplishes this.

Although the combination of machine learning and interior design has great potential for mining, it is limited by many practical factors such as the lack of building databases and data analogies, the functional limitations of computing machines, and the tight design time. This advanced technology is used in interior designing. It tends to take more time, resulting in few designers using it at work. However, with the replacement of computing functions and computing machines, the rapid development of artificial intelligence and the improvement of digital design databases, more and more designers will use programming and algorithms to solve design problems. Intelligent design solutions will also occupy a place in the design industry in the future.

RETRACTED

## Figures and Tables

**Figure 1:** McClam curve.

**Figure 2:** Traditional design firm workflow.

**Figure 3:** Modelling transfers to IFC information.

**Figure 4:** Processing of binarized drawing.

**Figure 5:** The generating principle of the interior design concept scheme.

**Figure 6:** The diagram of the Dong Xi Hu district map.

**Figure 7:** The diagram of the location of Dong Xi Hu procuratorate.

**Figure 8:** The diagram of building of Dong Xi Hu procuratorate.

**Figure 9:** Interior layout of the prosecutor's office.

**Figure 10:** Bubble chart of the interior layout.

**Figure 11:** Bubble chart of the new interior layout.

**Figure 12:** Transferred the new interior layout.

**Table 1:** The table of room types.

Numbers	Names of rooms	*Notes*
**1**	Relax spaces	*Special space*
**2**	Offices	*Basic space*
**3**	Coffee rooms	*Special space*
**4**	Meeting rooms	*Basic space*
**5**	Library	*Special space*
**6**	Elevator Hall	*Basic space*
**7**	Prosecutor's museum	*Special space*
**8**	Corridor	*Basic space*

**Table 2:** The table of room types.

Numbers	Link areas	Names of rooms
1	Corridor	Relax spaces
2	Corridor	Offices
3	Corridor and meeting room	Coffee rooms
4	Corridor and coffee rooms	Meeting rooms
5	Corridor	Library
6	Corridor	Elevator hall
7	Corridor	Prosecutor's museum
8	Relax spaces, offices, coffee rooms, meeting rooms, library, elevator hall, and prosecutor's museum	Corridor

## Data Availability

The datasets used in this study are available from the corresponding author on request.
